# The Increase in IL-1β in the Early Stage of Heatstroke Might Be Caused by Splenic Lymphocyte Pyroptosis Induced by mtROS-Mediated Activation of the NLRP3 Inflammasome

This article has been retracted.

**DOI:** 10.3389/fimmu.2019.02862

**Published:** 2019-12-11

**Authors:** Gong Wang, Tingting Shen, Ping Li, Zhen Luo, Yulong Tan, Genlin He, Xiaoliang Zhang, Ju Yang, Jun Liu, Yuan Wang, He Tang, Xue Luo, Xuesen Yang

**Affiliations:** ^1^Department of Tropical Medicine, College of Military Preventive Medicine, Army Medical University, Chongqing, China; ^2^Department of Neurology, Xinqiao Hospital, Army Medical University, Chongqing, China

**Keywords:** heatstroke, NLRP3 inflammasome, pyroptosis, mtROS, splenic lymphocytes

## Abstract

Interleukin-1β (IL-1β) is important for the pathological process of heatstroke (HS), although little is known regarding the main source of the IL-1β produced during the early stage of HS. In this study, heat stress led splenic lymphocytes to death with generation of inflammatory cytokines. The same phenomenon also occurs in animal models of heatshock. We observed that the death of splenic lymphocytes was identified to be pyroptosis. In addition, splenic lymphocyte pyroptosis can be induced by hyperpyrexia in a time- and temperature-dependent manner with NLR pyrin domain containing 3 (NLRP3) inflammasome activation. An NLRP3 inhibitor (MCC950) and a caspase-1 inhibitor (ac-YVAD-cmk) were used to confirm the role of the NLRP3/caspase-1 pathway in pyroptosis. With heat stress, levels of mitochondrial reactive oxygen species (mtROS) in splenic lymphocytes would significantly increase. Accordingly, the use of mtROS scavenger (Mito-TEMPO) could reduce the occurrence of pyroptosis and the activation of the NLRP3 inflammasome *in vitro*. In animal models of heatshock, Mito-TEMPO can inhibit activation of the NLRP3/caspase-1 pathway. Taken together, our data suggest that activation of the NLRP3 inflammasome mediates hyperpyrexia-induced pyroptosis in splenic lymphocytes. Perhaps one of the important initiators of pyroptosis is mtROS. Our data have elucidated a new molecular mechanism of IL-1β overexpression in the early stage of HS, providing a new strategy for IL-1β-targeted therapy in future clinical treatments for HS.

## Introduction

Specific mediators that lead to the occurrence of heatstroke (HS) and HS-related deaths are not clear, but previous studies have found that cytokines play an important role (1–3). These cytokines, including interleukin (IL)-1, are involved in the pathophysiology of HS. Regarding the specific role of the IL-1 family in the pathological process of HS, the relevant literature currently available is based only on circulating plasma levels in both HS patients and animal models. Clinical studies suggest that the degree of elevated IL-1 levels in the plasma of patients with HS is correlated with the degree of increase in body temperature (4–7). Animal experiments also suggest that high levels of IL-1β can be detected in both the plasma and central nervous system when the animal's core body temperature reaches HS (8–10). In the HS animal model, mice with HS would suffer from hypothermia (core temperature, Tc ≈ 29°C) during recovery. The trend of changes in the core body temperature with HS mice is consistent with changes in plasma IL-1β levels but does not match the level of change in IL-1α (11). Although IL-1β plays such an important role in the development of HS, we could not determine the source of the IL-1β that appears in the peripheral blood shortly after the onset of HS. Thus, understanding the source of IL-1β may provide important insights regarding not only the cause of the IL-1β increase but also the potential therapeutic benefits of HS treatment strategies targeting the source of IL-1β.

In the animal model of HS, the damage of organs did not occur simultaneously. As the pathological process of HS progresses, there is a significant difference in the time of injury of different organs (11, 12). Whether it is a clinical HS patient or an animal model of HS, there is no obvious liver damage at the time of HS onset. However, during the recovery period after HS, liver damage is a problem that needs to be focused on (12). Thus, spleen damage should occur earlier than liver damage. Since the spleen is the largest lymphatic organ, it contains a large number of immune cells, which could produce and respond to cytokines during inflammation. Therefore, we hypothesized that the spleen was the main source of the IL-1β produced during the early stage of HS.

How does the spleen produce IL-1β? The NLR pyrin domain containing 3 (NLRP3) inflammasome could regulate the activation of caspase-1, which promotes the maturation and secretion of cytokine precursors, such as pro-IL-1β and pro-IL-18 (13). There are five main types of inflammasome complexes that have been discovered, namely, NLRP1 inflammasome, NLRP3 inflammasome, NLRC4 inflammasome, IPAF inflammasome, and AIM2 inflammasome (14). The basic structure of most inflammatory vesicles consists of three parts: (1) NLR or ALR protein family as receptors; (2) ASC as adaptor; and (3) caspase as effector (15). Among them, the NLRP3 inflammasome is the best characterized. Activation of NLRP3 inflammasome promotes activation of caspase-1 to mediate cell swelling and cause cell death. The dead cells will have a plasma membrane rupture causing a large amount of proinflammatory components to be released (16). In addition to pathogen-associated molecular patterns (PAMPs), there are endogenous danger-associated molecular patterns (DAMPs) that could activate NLRP3 inflammasome (15, 17). Activation of NLRP3 will promote the activation of caspase-1, which in turn leads cells to pyroptosis. Pyroptosis is a new form of cell death depending on caspase-1 activation (18, 19). Therefore, we conclude that pyroptosis of splenic lymphocyte cells may be an important source of IL-1β.

Our results demonstrated that HS induced the NLRP3 inflammasome activation and subsequent pyroptosis in mouse splenic lymphocytes. Considering that HS induces NLRP3 activation through mitochondrial reactive oxygen species (mtROS) production under our experimental conditions, we demonstrated that NLRP3 inflammasome activation and pyroptosis were mediated by the increase in mtROS after HS. These data illustrate a new molecular mechanism of high IL-1β expression caused by HS, providing a new strategy for IL-1β-targeted therapy in future clinical treatments for HS.

## Materials and Methods

### Animals

This study was conducted according to the recommendations in the Guide for the Care and Use of Laboratory Animals. The protocol was approved by the Welfare and Ethics Committee of the Army Medical University. Male Institute of Cancer Research (ICR) mice (6–8 weeks old, 22–24 g) were obtained from the Animal Center of the Army Medical University (Chongqing, China). All animals were housed under standard laboratory conditions (12 h light/dark cycle, 23 ± 1°C, and 55 ± 5% humidity). The mice had free access to tap water and standard mouse diet at all times. The mice were acclimatized for 1 week before experiments.

### Treatment of Animals

#### Animal Models of Heatshock

To study the effects of heat stress on the spleen, the animals were assigned randomly to one of three groups (six mice per group). Core temperature (Tc) was monitored by an animal electronic thermometer (ALC-ET06; Alcbio, Shanghai, China) that was inserted 2 cm into the rectum. The mice in the control group were maintained at an ambient temperature of 23 ± 1°C. Mice in the HS 0 h and HS 3 h groups were exposed to 41 ± 0.5°C in the specific environmental control smart chamber (HOPE-MED 8150E, Tianjin, China) in the absence of food and water. Tc was measured at intervals of 10 min; when Tc > 42.5°C (HS onset), the mice were removed from the heat environment, weighed, and returned to the cage with *ad libitum* access to food and water for recovery at 25 ± 2°C. After 0 and 3 h of recovery from heat stress, the mice were anesthetized with an injection of sodium pentobarbital (40 mg/kg), and spleen tissues, kidney tissues, small intestine and large intestine tissues, and blood samples were immediately collected.

#### Inhibitor Administration

To confirm the role of mtROS and caspase-1 in splenic lymphocytes on the NLRP3/caspase-1 pathway in pyroptosis, we use Mito-TEMPO (mtROS inhibitor, 20 mg/kg, Santa Cruz Biotechnology, USA) dissolved in phosphate-buffered saline (PBS) and administered intraperitoneally 1 h before the high-temperature exposure; ac-YVAD-cmk (caspase-1 inhibitor, 6.5 mg/kg, Enzo Biochem, Inc., USA) dissolved in PBS containing 1% DMSO and injected 1 h before heat stress; and Z-DEVD-FMK (6.5 mg/kg, Sigma-Aldrich, USA) dissolved in PBS containing 1% DMSO and injected 1 h before heat stress.

### Cytokine Analysis

Blood samples were drawn from the right atrium after animals were anesthetized by a single intraperitoneal dose of sodium pentobarbital (40 mg/kg) and immediately separated. Cell supernatant was collected after heat stress. Those of IL-18, IL-1β, interferon (IFN)-γ, tumor necrosis (TNF)-α, IL-6, and IL-10 in serum and supernatant were measured using mouse enzyme-linked immunosorbent (ELISA) assay kits (Cloud-Clone Corp, Wuhan, China) according to the manufacturer's instructions. IL-12p70 in serum was measured using mouse ELISA assay kits (Abcam, Cambridge, MA), according to the manufacturer's instructions.

### Histology

Spleen and liver tissues were fixed in 10% neutral-buffered formalin, dehydrated, embedded in paraffin, and sliced to a thickness of 5 μm. Sections were subjected to hematoxylin–eosin (H&E) staining and then observed under an optical microscope (Bio-Rad, USA).

### Quantitative PCR

Total RNA was isolated from the spleen, kidney, small intestine, and colon by using an Eastep™ total RNA extraction reagent kit (Promega, LS1040, USA) according to the manufacturer's instructions. Complementary DNA (cDNA) was synthesized from 800 ng of total RNA using a PrimeScript™ RT reagent kit with gDNA Eraser (TaKaRa, RR047A, China). Real-time PCR was performed using a universal SYBR FAST qPCR kit (Kapa, KK4601, USA). Reactions were run in triplicate in a CFX96 real-time system (Bio-Rad, Hercules, CA, USA). The relative change in messenger RNA (mRNA) expression was calculated using the 2^−ΔΔCt^ method with HPRT as the endogenous standard for each sample.

### Western Blot Analysis

Protein extracts from the treated splenic lymphocyte cells and spleen of the experimental mice were collected using the radioimmunoprecipitation assay (RIPA) buffer (Beyotime, China) containing protease and phosphatase inhibitors (Roche, Penzberg, Germany). Then, 50 μg of the protein samples was separated using a 10% sodium dodecyl sulfate (SDS)–polyacrylamide gel electrophoresis (SDS-PAGE) and transferred to polyvinylidene fluoride (PVDF) membranes (Bio-Rad, CA, USA). The membranes were blocked for 1 h in 5% nonfat milk dissolved in PBS and then incubated with their respective primary antibodies against NLRP3 (1:1,000, AdipoGen), caspase-1 (1:1,000, AdipoGen), IL-1β (1:1,000, CST), gasdermin-D (GSDMD, 1:500; Biorbyt), and β-actin (1:1,000, Sigma) overnight at 4°C. The membranes were washed three times in Tris-buffered saline Tween-20 (TBST) and incubated with appropriate secondary antibodies conjugated to horseradish peroxidase (1:1,000, Sigma-Aldrich) for 1 h at room temperature. The bands were visualized with an enhanced chemiluminescence reagent (Bio-Rad) and were scanned and analyzed using a ChemiDoc MP gel imaging system (Bio-Rad).

### Splenic Lymphocyte Isolation

The primary splenic lymphocyte cells of male ICR mice were collected as follows: briefly, the mice were euthanized by an intraperitoneal injection of an overdose of sodium pentobarbital (50 mg/kg), and their bodies were then soaked in 75% ethanol. The spleen was removed and placed on a 200-μm pore mesh filter in a 35-mm dish, 5 ml of mouse lymphocyte separation medium (Dakewe, DKW33-R0400, China) was added to the dish, and the tissue was ground by means of a syringe piston. The suspension was immediately transferred to a centrifuge tube, covered with 1 ml of Roswell Park Memorial Institute (RPMI)-1640 medium (HyClone, USA), and then centrifuged at 800 × *g* for 30 min. The cell pellet was resuspended with 10 ml of RPMI-1640 and washed at room temperature. After centrifugation at 800 × *g* for 10 min, the cell pellet was resuspended in RPMI-1640 medium, and the cells were counted. Specific details of splenic lymphocyte isolation and purity of harvested cells are shown in Supplementary Figure 1.

### Cell Culture and Treatment

The isolated cells were seeded at a density of 1 × 10^6^ cells per well in a six-well plate in RPMI-1640 with 10% fetal bovine serum (HyClone, UT, USA), 100 U/ml of penicillin, and 100 μg/ml of streptomycin (Beyotime, China) at 37°C and 5% CO_2_. Cells were grown to 80–90% confluence. For heat stress treatments, culture dishes were placed into incubators with different temperatures (39 ± 0.5°C, 41 ± 0.5°C, and 43 ± 0.5°C) for different times (0, 15, 30, 45, and 60 min) and a culture humidity >90%. Control cells were maintained in incubators at 37 ± 0.5°C.

To block caspase-1, the caspase-1 inhibitor AC-TYR-VAL-ALA-ASP-chloromethylketone (ac-YVAD-cmk) (0.3 mg/ml; Enzo Biochem, Inc., New York, USA) was added to the cells for 30 min before heat stress. MCC950 is a specific inhibitor of NLRP3, and MCC950 (50 μM, MedChemExpress, Shanghai, China) dissolved in normal saline was given 1 h before heat stress *in vitro*. Z-DEVD-FMK (3 μM, Sigma-Aldrich, USA) as the specific caspase-3 inhibitor was added to the cells 1 h before heat stress. In some experiments, the antioxidant *N*-acetyl cysteine (NAC, Beyotime, 5 mM) and the mitochondria-targeted antioxidant Mito-TEMPO (1 μM, Santa Cruz Biotechnology) were added to the cells before heat stress.

### Determination of Splenic Lymphocyte Pyroptosis

A FAM-FLICA caspase-1 detection kit (ImmunoChemistry, Bloomington, MN, USA) was used to assess pyroptotic cell death in splenic lymphocytes isolated from the mouse spleens. After different treatments of primary splenic lymphocytes subsequently stained with caspase-1 and SYTOX™ Green Nucleic Acid Stain (SYTOX Green), cells that were double positive for active caspase-1 and SYTOX Green staining were identified, and the cells were analyzed on a flow cytometer.

### LDH Release Assay

Splenic lymphocyte cells were seeded in sterile 96-well culture plates at a density of 8 × 10^3^ cells per well. Lactate dehydrogenase (LDH) was detected using the Cytotoxicity Detection Kit Plus LDH (Roche, USA), and the supernatants were used to assess LDH activity according to the manufacturer's protocol.

### Determination of Splenic Lymphocyte Oxidative Stress

The total intracellular reactive oxygen species (ROS) induced by heat stress after antioxidant treatment was measured in primary splenic lymphocytes. The cells were incubated for 20 min with the fluorescent probe dichlorodihydrofluorescein diacetate (DCFH-DA) (Beyotime, China) at 37°C. The fluorescence was detected on a flow cytometer. The mtROS level was measured using a MitoSOX Red superoxide indicator (Molecular Probes™, USA) according to the manufacturer's protocol. Briefly, cells were labeled with 5 μM of a MitoSOX™ reagent working solution for 10 min at 37°C, protected from light, and then washed gently three times with warm Hank's balanced salt solution with calcium and magnesium [HBSS/Ca/Mg, Gibco (14025-092)]. The stained cells were imaged on a fluorescence inverted microscope (Bio-Rad). The intensity of mtROS was measured using the ImageJ software.

### Statistical Analysis

Statistical analyses were performed by using the SPSS software. Each experiment was repeated a minimum of three times to ensure the repeatability of the findings. Data are expressed as the mean ± SEM. One- or two-way analysis of variance (ANOVA) followed by Tukey's test was used for comparisons between groups. Statistical significance was established at *p* < 0.05, unless otherwise indicated.

## Results

### HS-Induced Spleen Injury and Inflammatory Cytokine Upregulation

In previous studies, the histological damage in the spleen was detected during the low-temperature period, and this study intends to explore the source of IL-1β in the early stage of HS. Therefore, we have set the observation time of the animal model to 0 h (high-body-temperature period when out of the chamber) and 3 h (low-body-temperature period). Figure 1A shows histological changes in the spleen after HS. At the time of HS (0 h), the body temperature was high (Tc = 43°C), the spleen sinus expanded, and the red pulp region showed obvious congestion, but no obvious cell damage and changes were observed. Three hours after the occurrence of HS (low-body-temperature period, Tc = 29°C), the splenic sinus congestion was severe, and lymphocyte disintegration led to increased cell debris in the red pulp and phagocytosis by phagocytic cells.

**Figure 1:** Heatstroke (HS) induced spleen injury and inflammatory cytokine upregulation. **(A)** Representative pathological images of the spleen from sham heated mice (left) and HS mice (0 h, middle; 3 h, right) stained with H&E at a magnification of ×100. At the time of HS (0 h), the body temperature was high (Tc = 43°C), the spleen sinus expanded, and the red pulp region showed obvious congestion (black arrow), but no obvious cell damage and changes were observed. Three hours after the occurrence of HS (low-body-temperature period, Tc = 29°C), the splenic sinus congestion was severe (black arrow), and lymphocyte disintegration led to increased cell debris in the red pulp and phagocytosis by phagocytic cells. In each group, *n* = 6. H&E, hematoxylin and eosin. **(B–E)** Interleukin (IL)-1β and IL-18 protein expression in serum **(B,C)** measured by enzyme-linked immunosorbent assay (ELISA) at the time point of HS onset (0 h) and 3 h after onset. Meanwhile, the spleen **(D,E)** was measured by real-time quantitative PCR at the time point of HS onset (0 h) and 3 h after onset. Means and standard deviations are shown, *n* = 6 per group, ^*^p < 0.05 compared with the sham heated group, ^**^p < 0.001 compared with the sham heated group.

In order to further confirm that the spleen is the injured organ in the early stage of HS among important organs, we also observed the liver in the pathological observation of the spleen. Under our experimental conditions, at the time of HS (0 h), the body temperature was high (Tc = 43°C), the hepatic sinus is dilated, and some areas of the section are visible with congestion. Three hours after the occurrence of HS (low-body-temperature period, Tc = 29°C), the slice shows visible sinusoidal dilatation. Neutrophils and mononuclear cells are seen in some areas. The basic structure of liver tissues is relatively intact (Supplementary Figure 2).

The serum IL-1β and IL-18 protein concentrations (Figures 1B,C) began to increase immediately after the onset of HS (0 h), but the change was not statistically significant (*p* = 0.182). There was a significant increase at 3 h (low body temperature) (*p* = 0.025). In spleen tissues, we examined the expression of IL-1β and IL-18 mRNA (Figures 1D,E). The mRNA expression levels of IL-1β and IL-18 were high immediately after the occurrence of HS (0 h) but decreased at 3 h (lower body temperature). The changes in serum IL-1β and IL-18 protein concentrations were consistent with the pathological changes in the spleen.

At the same time, we also evaluated the expression of IL-12p70, IFN-γ, TNF-α, IL-6, and IL-10 in serum. Among them, IL-12p70, IFN-γ, and TNF-α did not show statistically significant changes at the evaluated phase points (Figures 2A–C). IL-6 showed an upregulation of expression at the onset of HS (0 h, high body temperature), which was significantly increased at 3 h (lower body temperature) after HS (159.1 ± 53.8 pg/ml; *p* < 0.01) (Figure 2D). The expression trend of IL-10 was consistent with the IL-6 pattern (Figure 2E).

**Figure 2:** Changes in serum of IL-12p70 **(A)**, IFN-γ **(B)**, TNF-α **(C)**, IL-6 **(D)**, and IL-10 **(E)** in mice following heatstroke. The blood samples were obtained at 0 and 3 h after the onset of heatstroke from heatstroke mice. Messenger RNA (mRNA) expression of cytokines **(F–J)**. Spleen tissue was collected at 0 and 3 h after heatstroke from heatstroke mice. The expression of **(F)** IL-12p70, **(G)** IFN-γ, **(H)** TNF-α, **(I)** IL-6, and **(J)** IL-10 was measured using real-time RT-PCR. Values are shown as means ± SEM for three independent experiments, *n* = 6–8 per group, ^*^p < 0.05, ^**^p < 0.01. IL-12p70 indicates interleukin-12p70; IFN-γ indicates interferon gamma; TNF-a indicates tumor necrosis factor alpha; IL-6 indicates interleukin-6; and IL-10 indicates interleukin-10.

At last, splenic cytokine mRNAs were analyzed by reverse-transcription real-time PCR. As shown in Figures 2F–J, the synthesized levels of IL-12p70, IFN-γ, and TNF-α mRNAs were significantly increased in the spleen tissues of HS mice compared with the same tissues taken from the control group at 0 and 3 h after HS. TNF-α mRNA expression was significantly increased, but it was not sustained. In the process of increasing, a stage of lower expression was noted at 3 h. IL-6 mRNA expression decreased and then increased, but 3 h (lower body temperature) after HS, it still has a significant increase.

### HS-Induced NLRP3 Inflammasome Activation and Pyroptosis in Splenic Lymphocytes *in vivo*

Consistent with the previous findings, a high expression of IL-1β and IL-18 was observed in the peripheral blood and spleen tissues of mice under hypothermia, and IL-1β is the most widely recognized downstream product of NLRP3 inflammatory bodies. Therefore, we wanted to explore whether NLRP3 inflammatory corpuscles are involved in the spleen damage caused by heat stress. We examined the gene and protein expression of NLRP3 in the spleen of mice with heat-induced disease and found increased gene and protein of NLRP3 in the high-temperature period (0 h) and the lower body temperature (3 h) (Figures 3A,B). A western blot (WB) assay showed that the expression level of caspase-1 increased at 0 and 3 h after the end of heat stress (Figure 3C).

**Figure 3:** Heatstroke induced splenic lymphocyte NLRP3 inflammasome activation and pyroptosis *in vivo*. Gene **(A)** and protein **(B)** expression of NLR pyrin domain containing 3 (NLRP3) in the spleen of a mouse heatstroke model. **(C)** Effect of heatstroke induce cleaved caspase-1 (Casp1 p20) measured by western blot. **(D)** Immunoblotting analysis of cleaved gasdermin-D (GSDMD) in the spleen proves whether pyroptosis was activated at 0 and 3 h after the end of heatstroke. **(E)** Membrane pore formation (SYTOX Green staining, horizontal) and caspase-1 activation (FLICA 660-YVAD-FMK staining, vertical) measured by flow cytometry. Values are mean ± SD for three independent experiments and *n* = 6. ^*^p < 0.05, ^**^p < 0.01 compared with the sham heated group.

The recent research shows that protein GSDMD as the marker of pyroptosis happened. When active caspase-1 or caspase-11 enzymatically cleaves GSDMD into two fragments, GSDMD-N will disrupt cell membrane and induce pyroptosis. Here, we examined the protein expression of GSDMD *in vivo* and found that 0 and 3 h after the end of heat stress, there was an increase in cleaved GSDMD in the spleen (Figure 3D), which means that pyroptosis was activated in HS.

Cells undergoing pyroptosis are usually thought to be double positive for caspase-1 and SYTOX Green staining. To determine whether the loss of spleen cell membrane integrity leads to pyroptosis, we isolated spleen mononuclear cells from a mouse model of HS and then detected activated caspase-1 and SYTOX Green staining double-positive cells with flow cytometry. As shown in Figure 3E, the ratio of caspase-1 and SYTOX Green staining double-positive cells increased at 0 h (high body temperature) after HS and increased significantly at 3 h (low body temperature) (*p* < 0.01 compared with the control group).

### Heat Stress-Induced Splenic Lymphocyte Pyroptosis *in vitro*

To further clarify that HS can induce splenic lymphocyte death, in addition to *in vivo* experimental studies, we also isolated splenic lymphocytes for *in vitro* experiments. In order to confirm the conditions where heat stress induced splenic lymphocyte pyroptosis *in vitro*, in subsequent studies, splenic lymphocytes were placed into incubators with different temperatures (37 ± 0.5°C, 39 ± 0.5°C, 41 ± 0.5°C, and 43 ± 0.5°C) for different times (0, 15 min, 30, 45, and 60 min), and cell viability was determined using the Cell Counting Kit-8 (data not shown). When splenic lymphocytes were exposed with 39, 41, or 43°C, cell viability is inversely related to temperature. These results indicate that heat stress induced significant cell death in splenic lymphocyte in a dose- and time-dependent manner. Based on the results of cell viability, cells cultured at 43°C for 60 min will bring systematic errors to the results.

According to the literature, pyroptosis lead to cell lysis by destroying cell membrane integrity. To determine the effect of heat stress on the cell membrane integrity of splenic lymphocytes, the activity of LDH in the supernatant was measured. Cells were incubated at different temperatures (37, 39, 41, and 43°C) for 45 min. When the cells were cultured with ambient temperature 41°C, the LDH activity was increased (*p* < 0.05). When the cells were cultured with ambient temperature 43°C, the LDH activity was significantly increased (*p* < 0.01) (Figure 4A). Cells were subjected to heat stress (43°C) for different times (0, 15, 30, and 45 min). The LDH activity began to significantly increase after 30 min cultured at 43°C. Moreover, LDH activity increased significantly with the prolongation of culture time (*p* < 0.01) (Figure 4B).

**Figure 4:** Heat stress destroyed cell membrane integrity of splenic lymphocytes *in vitro*. **(A)** Cells were incubated at different temperatures (37, 39, 41, and 43°C) for 45 min. Levels of lactate dehydrogenase (LDH) release are shown in the bar graph. **(B)** Cells were subjected to heat stress (43°C) for different times (0, 15, 30, and 45 min). Levels of LDH release are shown in the bar graph. **(C)** Cells were incubated at 37°C (control) and at different temperatures (39, 41, and 43°C) for 45 min; effects of different temperatures on the caspase-1 (FLICA 660-YVAD-FMK staining, vertical) and SYTOX Green (horizontal) double-positive cells measured by flow cytometry. The ratio of caspase-1 and SYTOX Green double-positive cells is shown in the bar graph. **(D)** Cells were subjected to heat stress (43°C) for different times (0, 15, 30, and 45 min). Effects of different durations on caspase-1 (FLICA 660-YVAD-FMK staining, vertical) and SYTOX Green (horizontal) double-positive cells under high temperature measured by flow cytometry. The ratio of caspase-1 and SYTOX Green double-positive cells is shown in the bar graph. Values are mean ± SD for six independent experiments. ^*^p < 0.05, ^**^p < 0.01 compared with the control group (37°C) or sham heated group.

To determine whether death of splenic lymphocytes in response to heat stress are due to pyroptosis, we measured active caspase-1 and SYTOX Green staining double positivity in splenic lymphocytes via flow cytometry. After the cells were cultured at different temperatures (37, 39, 41, and 43°C) for 45 min, the ratio of caspase-1 and SYTOX Green staining double-positive cells began to increase at 41°C. When the cells were cultured with ambient temperature 43°C, the ratio of caspase-1 and SYTOX Green staining double-positive cells was significantly increased (*p* < 0.01) (Figure 4C). Cells were subjected to heat stress (43°C) for different times (0, 15, 30, and 45 min). The ratio of caspase-1 and SYTOX Green staining double-positive cells began to increase after 30 min cultured at 43°C. Moreover, the ratio increased significantly with the prolongation of culture time (*p* < 0.01) (Figure 4D).

To verify that cell death caused by heat stress is caused by pyroptosis, we used a NLRP3 inhibitor (MCC950), caspase-1 inhibitor (ac-YVAD-cmk, YVAD), and caspase-3 inhibitor (Z-DEVD-FMK). MCC950 is effective in blocking the NLRP3 inflammasome. YVAD is effective in blocking the cleavage of caspase-1 caused by heat stress and the subsequent maturation of IL-1β. Cells were subjected to heat stress (37 and 43°C) for 45 min, with or without the NLRP3 inhibitor (MCC950), caspase-1 inhibitor (YVAD), and caspase-3 inhibitor (DEVD). When the cells were cultured with ambient temperature 43°C, the LDH activity was significantly increased (*p* < 0.01). MCC950 and YVAD could significantly reduce the release of LDH in response to heat stress (*p* < 0.01), while DEVD only slightly reduce the release of LDH, there was no statistical difference in this change. The flow cytometry results showed that heat stress significantly increased the ratio of caspase-1 and SYTOX Green staining double-positive cells, whereas the ratio of double-positive cells significantly decreased with MCC950 and YVAD pretreatment heat stress (*p* < 0.01), DEVD could reduce the ratio of caspase-1 and SYTOX Green staining double-positive cells, but there is no statistical difference (Figure 5).

**Figure 5:** MCC950 or ac-YVAD-cmk reduces the damage of cell membrane integrity of spleen lymphocytes induced by heat stress *in vitro*. Cells were subjected to heat stress (37 and 43°C) for 45 min, with or without the NLR pyrin domain containing 3 (NLRP3) inhibitor (MCC950), caspase-1 inhibitor (YVAD), and caspase-3 inhibitor (DEVD). Levels of lactate dehydrogenase (LDH) release are shown in the bar graph. Membrane pore formation (SYTOX Green staining, horizontal) and caspase-1 activation (FLICA 660-YVAD-FMK staining, vertical) measured by flow cytometry. The ratio of caspase-1 and SYTOX Green double-positive cells is shown in the bar graph. Values are mean ± SD for six independent experiments. ^*^p < 0.05, ^**^p < 0.01 compared with the sham heated group (43°C).

### Heat Stress Activates the NLRP3/Caspase-1 Pathway in Splenic Lymphocytes *in vitro*

We assessed the activation of NLRP3 by measuring the levels of NLRP3, caspase-1, and IL-1β. After the cells were cultured at different temperatures (37, 39, 41, and 43°C) for 45 min, the NLRP3, caspase-1, and IL-1β protein expression was increased with the change of temperatures. When the cells were cultured with ambient temperature 41°C, the NLRP3, caspase-1 and IL-1β protein expression was significantly increased (*p* < 0.01). Cells were subjected to heat stress (43°C) for different times (0, 15, 30, and 45 min). The NLRP3, caspase-1, and IL-1β protein expression was increased with the prolongation of culture time. When the heating time reaches 30 min, the NLRP3, caspase-1, and IL-1β protein expression began to significantly increase (*p* < 0.01) (Figure 6).

**Figure 6:** Effect of heat stress on NLR pyrin domain containing 3 (NLRP3), caspase-1, and interleukin-1β (IL-1β) protein expression. **(A)** Cells were incubated at different temperatures (37, 39, 41, and 43°C) for 45 min. NLRP3, caspase-1, and IL-1β were measured by western blot. **(B)** Cells were subjected to heat stress (43°C) for different times (0, 15, 30, and 45 min). NLRP3, caspase-1, and IL-1β are measured by western blot. Levels of NLRP3, caspase-1, and IL-1β protein expression are shown in the bar graph. Values are mean ± SD for six independent experiments. ^*^p < 0.05, ^**^p < 0.01 compared with the control group (37°C) or sham heated group.

### mtROS Involved in Heat Stress-Induced NLRP3 Activation and Pyroptosis in Splenic Lymphocytes

ROS is involved in the activation of NLRP3 inflammatory bodies. It has been reported that mtROS play a critical role in the activation of NLRP3. To determine whether mtROS play an important role in heat stress-induced NLRP3 inflammatory body activation in splenic lymphocytes, we examined mtROS and intracellular ROS levels, as well as specific inhibitors of mtROS and intracellular ROS. To observe the effect of mtROS and ROS removal on NLRP3 inflammatory body activation, we used *in vitro* experiments cells were incubated at different temperatures (37, 39, 41, and 43°C) for 45 min. When the cells were cultured with ambient temperature 41°C, the intracellular ROS and mtROS levels were increased (*p* < 0.05). When the cells were cultured with ambient temperature 43°C, the intracellular ROS levels and mtROS were significantly increased (*p* < 0.01) (Figures 7A,C). The heat stress temperature of the cell culture was still set at 43°C, and the heat treatment times were 0, 15, 30, and 45 min. It was found that heat stress promoted intracellular ROS levels and mtROS production in a time-dependent manner (Figures 7B,D).

**Figure 7:** Effect of heat stress on intracellular reactive oxygen species (ROS) and mitochondrial ROS. **(A,C)** Cells were incubated at different temperatures (37, 39, 41, and 43°C) for 45 min. **(B,D)** Cells were subjected to heat stress (43°C) for different times (0, 15, 30, and 45 min). Intracellular ROS were analyzed in **(A,B)**. Mitochondrial ROS were analyzed in **(C,D)**. Levels of intracellular ROS and mitochondrial ROS are shown in the bar graph. Values are mean ± SD for six independent experiments. ^**^p < 0.01 compared with the control group (37°C) **(A,C)** or sham heated group **(B,D)**.

Inhibition of mtROS was performed using a mtROS-specific scavenger (Mito-TEMPO), and total ROS inhibition was achieved with a scavenger (NAC). Splenic lymphocytes were pretreated with Mito-TEMPO or NAC and then subjected to heat stress. Pretreatment with Mito-TEMPO or NAC was able to significantly inhibit the NLRP3, caspase-1, and GSDMD activation induced by heat stress and the production of mature IL-1β in cells (*p* < 0.01) (Figures 8A–F). To make clear the role of mtROS in heat stress-induced pyroptosis, we examined the ratio of caspase-1 and SYTOX Green double-positive cells after treatment with Mito-TEMPO or NAC. As shown in Figure 9, Mito-TEMPO and NAC were able to significantly reduce heat stress-induced cell pyroptosis at 43°C (*p* < 0.01).

**Figure 8:** Effects of different reactive oxygen species (ROS) scavengers on the levels of NLR pyrin domain containing 3 (NLRP3), caspase-1, gasdermin-D (GSDMD), and interleukin-1β (IL-1β) proteins under heat stress. Cells were subjected to heat stress (43°C) for 45 min with or without ROS scavengers [Mito-TEMPO or *N*-acetyl cysteine (NAC)]. **(A**–**E)** NLRP3, caspase-1, GSDMD, and IL-1β were measured by western blot. Levels of NLRP3, caspase-1, GSDMD, and IL-1β protein expression are shown in the bar graph. **(F)** IL-1β protein expression in cell supernatants measured by enzyme-linked immunosorbent assay (ELISA). Values are mean ± SD for six independent experiments. ^**^p < 0.01 compared with the control group (37°C). ##*p* < 0.01, compared with the heat group (43°C).

**Figure 9:** Mitochondrial reactive oxygen species (ROS) mediate heat stress-induced pyroptosis in splenic lymphocytes *in vitro*. **(A)** Cells were subjected to heat stress (43°C) for 45 min with or without ROS scavengers [Mito-TEMPO or *N*-acetyl cysteine (NAC)]. In the other groups, cells were incubated at 37°C and treated with Mito-TEMPO or NAC or YVAD. Representative flow cytometry results of TEMPO and NAC on heat stress-induced double positivity for caspase-1 (vertical) and SYTOX Green (horizontal). **(B)** Quantification of the membrane pore formation (SYTOX Green staining, horizontal) and caspase-1 activation cells was calculated from **(A)**. Values are mean ± SD for six independent experiments. ^**^p < 0.01 compared with the control group at 37°C. ##*p* < 0.01, compared with the control group at 43°C.

Since in *in vitro* experiments, inhibition of mtROS has a significant effect on the heat stress-induced pyroptosis, we further verified this through *in vivo* experiments, hoping that the exploration of basic research can be transformed into clinical applications. For *in vivo* experiments, we use Mito-TEMPO dissolved in PBS and administered intraperitoneally to mice before heat stress. NLRP3, caspase-1, GSDMD, and IL-1β in the sham heated group are significantly increased (*p* < 0.01), while with a mtROS-specific scavenger (Mito-TEMPO), there were a significant reduction in NLRP3 and caspase-1 and a reduction in lysed GSDMD and IL-1β (*p* < 0.05) (Figure 10).

**Figure 10:** The effect of Mito-TEMPO on heat stress-induced pyroptosis *in vivo*. Mice with or without Mito-TEMPO (20 mg/kg) before heat stress; then spleen tissues were separated from mice 3 h after heatstroke. NLR pyrin domain containing 3 (NLRP3), caspase-1, gasdermin-D (GSDMD), and interleukin-1β (IL-1β) protein expression in spleen tissues measured by immunoblotting. Levels of NLRP3, caspase-1, GSDMD, and IL-1β protein expression are shown in the bar graph. Means and standard deviations are shown; results are representative of three separate independent experiments, *n* = 6 per group, ^**^p < 0.01 compared with the control group (37°C), #*p* < 0.05, ##*p* < 0.01 compared with the sham heated group.

To confirm the role of caspase-1 in splenic lymphocytes on the NLRP3/caspase-1 pathway in pyroptosis *in vivo*, we use YVAD (caspase-1 inhibitor) and DEVD (caspase-3 inhibitor) dissolved in PBS containing 1% DMSO and injected 1 h before heat stress. Caspase-1 and IL-1β significantly increased in the sham heated group (*p* < 0.01). Pretreatment with YVAD was able to significantly inhibit caspase-1 activation induced by heat stress (*p* < 0.01); DEVD has little influence. Pretreatment with YVAD and DEVD could obviously decrease the production of mature IL-1β (*p* < 0.01) (Figure 11).

**Figure 11:** YVAD inhibited NLR pyrin domain containing 3 (NLRP3)/caspase-1-dependent pyroptosis and inflammatory cytokines in heatstroke mice. Mice were treated with YVAD [caspase-1 inhibitor, 6.5 mg/kg, in 1% DMSO in phosphate-buffered saline (PBS)] and DEVD (caspase-3 inhibitor, 6.5 mg/kg, in 1% DMSO in PBS) injected 1 h before heat stress. Spleen tissues were isolated from mice 3 h after heatstroke. Proteins were obtained, and representative western blot and quantitative analyses of the protein level of caspase-1 and interleukin-1β (IL-1β) in spleen tissues were performed. Means and standard deviations are shown; results are representative of three separate independent experiments, *n* = 6 per group, ^**^p < 0.01 compared with the control group (37°C), ##*p* < 0.01 compared with the sham heated group.

## Discussion

The purpose of this study was to clarify the source of high IL-1β levels in plasma at HS onset. Based on our results, high IL-1β levels in plasma might come from pyroptotic cells of splenic lymphocytes in a mouse HS model. The presence of pyroptotic cell death was due to hyperpyrexia with hyperactivation of the NLRP3 inflammasome. The occurrence of pyroptosis was defined by the positive results for both active caspase-1 and SYTOX Green. Moreover, both a caspase-1 inhibitor (Z-YVAD-FMK) and a NLRP3 inhibitor (MCC950) reduce cell death caused by heat stress. Pyroptosis will lead to a high level of IL-1β production, which might be an important source of IL-1β in the early stage of HS.

There are two main methods for HS animal model: (1) animal with anesthesia and (2) animals with an awake state. Anesthetics have a protective effect on the nervous system of animals with cerebral ischemia or metabolism. More importantly, animals under anesthesia will lose their bodies' ability to regulate their body temperature. The awake-animal model is closer to the physiological state and is more suitable for the pathophysiology of HS. Therefore, we use animals in conscious state for research. Animal ethics stipulates that some animals are forbidden to be used as a HS model in the waking state, such as rabbits, dogs, and baboons. In animal models of HS, mice and rats are the main source. In the authors' previous studies of HS, mice were used as animal models. For the completeness and correspondence of the experimental results, this study continued to use mice to establish a HS animal model. For heat tolerance, studies have found that estrogen and progesterone have protective effects on central and peripheral nerve injury caused by HS. Therefore, we believe that males are more suitable for the establishment of thermal radiation models.

In HS research using mice as animal models, 101 articles were searched through Web of Science. American scholars have published the most articles on the study of HS. Among these articles, there are many studies that focus on exertional HS. The exertional HS model is significantly different from the classic HS model used in our manuscript. Animal models similar to our study have been the most studied by scholars in Taiwan. The type of mouse commonly used by Taiwanese scholars is ICR mice. In order to have a better correspondence with peer studies, our study used ICR mice.

Although the spleen is the largest immune organ, it has not received much attention in terms of the pathogenesis of HS. Little is known about the role of the spleen in the HS process. Leon et al. used pathological sections to observe pathological changes in eight important organs (the kidney, spleen, liver, brain, heart, lung, small intestine, and large intestine) in a mouse model of HS. Under their experimental conditions, only three organs were sensitive to hyperthermia, namely, the kidney, spleen, and small intestine. There was no obvious change in the liver, brain, heart, lung, and large intestine in pathological sections. Histological damage to the spleen is detected during hypothermia and precedes the damage in other important organs (such as the liver) (11). In addition, the expression of IL-1β and IL-18 genes in the spleen reached the peak value as early as Tc, max (HS onset) (20). In our study, we found that pyroptosis occurred in splenic lymphocytes in the early stage of HS. The pyroptosis of spleen cells may be an important mechanism of hyperthermia-induced splenic pathological damage. Splenic damage was detected immediately after hypothermia, and the number of lesions decreased within 24 h of recovery. Lymphoid necrosis was observed in the white pulp of the spleen, as characterized by small clusters of nuclear and cellular debris that each occurred within a tingible body macrophage (11). The white pulp of the spleen is located around the small arterioles in the spleen and consists of two parts: the outer side band containing B cells and CD4^+^ T cells and the inner lymphatic sheath surrounding the blood vessels. We will probably explore the fraction of lymphocytes in the white pulp that undergo pyroptosis.

Pyroptosis is a caspase-1-dependent programmed cell death with plasma membrane rupture, and proinflammatory release (21–24). Su et al. have reported that hyperthermia can cause liver cell pyroptosis, which may be an indirect effect of heat stress on liver injury (25). However, the role of pyroptosis in the acute spleen injury caused by HS has not been explored. Our study demonstrates that hyperthermia could cause pyroptosis of splenic lymphocytes. We found that splenic lymphocyte pyroptosis is dependent on NLRP3 inflammasome activation. Hyperthermia-induced pyroptosis in splenic lymphocytes could be reduced by the NLRP3 inhibitor (MCC950) and caspase-1 inhibitor (YVAD), but the caspase-3 inhibitor (DEVD) could not do it. The results suggest that hyperthermia can activate inflammasomes in splenic lymphocytes and lead to pyroptosis. Because lymphocytes need stimulation to proliferate, small interfering RNA (siRNA) silencing of target genes cannot be performed on primary splenic lymphocytes. Thus, we were unable to knock down NLRP3 protein to assess its role in hyperthermia-induced lymphocyte pyroptosis. NLRP3-knockout mice should be used to investigate the role of NLRP3 protein in hyperthermia-induced lymphocyte pyroptosis. In our study, we used closed colony animals (ICR mice). The genetic composition of animals in closed populations is highly heterozygous and has a genetic heterogeneity similar to that of humans. Unfortunately, no knockout model with closed colony mice can be used.

It was found that hyperthermia can induce proinflammatory cytokine production in different tissues and cells (3). The mechanism by which hyperthermia leads to inflammation is still unknown. Pyroptosis relies on the activation of caspase-1, which cleaves the proinflammatory cytokine precursors pro-IL-1β and pro-IL-18 into their mature forms (26, 27). Pyroptosis would lead to leakage of cytosolic contents (DAMPs), causing abundant proinflammatory cytokine production (28). The occurrence of pyroptosis is therefore essentially proinflammatory. Our study found that the hyperthermia-induced pyroptosis of splenic lymphocytes may be one of the important mechanisms of inflammation in HS. It is worth mentioning that although we detected pyroptosis of splenic lymphocytes and high levels of proinflammatory cytokines, such as IL-1β, IL-18, and IL-6, some important proinflammatory factors, such as IL-12p70, IFN-γ, and TNF-α, were not upregulated at the time points we observed. IL-12p70 is a protein that is very sensitive to pathological stimuli (29). In mice with HS, intestinal damage occurs at Tc, max (HS onset), and endotoxin may have entered the peripheral blood. In the hypothermia period, the spleen, the small intestine, and the kidneys have already undergone pathological changes. However, we did not detect significant changes in IL-12p70 in blood samples at hypothermia and Tc, max (HS onset), contrary to our expectations. Pyroptosis can trigger inflammation, but not all inflammatory cytokines are triggered by pyroptosis. In future studies, we will continue to explore whether the levels of inflammatory factors such as IL-12p70, IFN-γ, and TNF-α will change during a longer recovery period and explore the initiating factors for these changes.

ROS production is one of the possible mechanisms of NLRP3 inflammasome activation (15). Recent studies have found that mtROS production appears to play a key role in NLRP3 inflammasome activation (30). Some scientists have confirmed that heat stress can produce ROS (31, 32). In our study, stimulation with hyperthermia resulted in the accumulation of both intracellular ROS and mtROS in splenic lymphocytes. The inhibition of mtROS would block the NLRP3, caspase-1 activation, IL-1β maturation, and cleaved GSDMD. Moreover, to inhibit mtROS could reduce the pyroptosis in splenic lymphocytes. For verification, *in vivo* experiments were performed, where we were able to achieve the same result. Thus, we believe that mtROS plays an important role in NLRP3 inflammasome activation. Of course, this study does not rule out the possible mechanisms of NLRP3 inflammasome activation, including potassium efflux, lysosomal destabilization, and the release of lysosomal cathepsins (33–36) Further investigation into the upstream mechanisms involved in hyperthermia-triggered NLRP3 inflammasome activation in splenic lymphocytes is needed.

In conclusion, our study found that hyperthermia could induce caspase-1-dependent pyroptosis and inflammation in splenic tissues. Although the spleen is the largest immune organ and is sensitive to hyperthermia, it has received less attention than expected regarding the pathogenesis of HS. We demonstrated that hyperthermia-induced pyroptosis in splenic lymphocytes is caused by the NLRP3 inflammasome activation. Moreover, mtROS generation is one of the upstream mechanisms involved in hyperthermia-triggered NLRP3 inflammasome activation and pyroptosis. Our study has elucidated a new molecular mechanism underlying IL-1β overexpression in the early stage after HS, providing a new strategy for IL-1β-targeted therapy in future clinical treatments for HS.

## Data Availability Statement

All datasets generated for this study are included in the article/Supplementary Material.

## Ethics Statement

The animal study was reviewed and approved by the Welfare and Ethics Committee of Army Medical University.

## Author Contributions

GW, PL, and TS wrote the manuscript, contributed to the analyses, and incorporated coauthors' edits and feedback into the final version of the manuscript. YT, GH, and ZL co-wrote the manuscript. PL, TS, YT, ZL, YW, and HT performed the experiments. XZ, JY, and JL conducted the analyses. XL and XY conceived the experiments and provided funding, design, overall supervision for this study and have assumed responsibility for keeping the coauthors informed of this manuscript's progress through the editorial review process, the content of the reviews, and any revisions made. All of the authors listed have agreed to the submission of the manuscript in this form.

### Conflict of Interest

The authors declare that the research was conducted in the absence of any commercial or financial relationships that could be construed as a potential conflict of interest.
